The article "Protective Effects of Amauroderma rugosum on Doxorubicin-Induced Cardiotoxicity through Suppressing Oxidative Stress, Mitochondrial Dysfunction, Apoptosis, and Activating Akt/mTOR and Nrf2/HO-1 Signaling Pathways" was retracted in 2023. Reasons: signs of a paper mill; compromised peer review; unreliable results or conclusions.

# Protective Effects of *Amauroderma rugosum* on Doxorubicin-Induced Cardiotoxicity through Suppressing Oxidative Stress, Mitochondrial Dysfunction, Apoptosis, and Activating Akt/mTOR and Nrf2/HO-1 Signaling Pathways

**DOI:** 10.1155/2022/9266178

**Published:** 2022-06-01

**Authors:** Jingjing Li, Yanfen Cheng, Renkai Li, Xiaoping Wu, Chengwen Zheng, Polly Ho-Ting Shiu, Jacqueline Cho-Ki Chan, Panthakarn Rangsinth, Conghui Liu, Susan Wai-Sum Leung, Simon Ming-Yuen Lee, Chen Zhang, Chaomei Fu, Jinming Zhang, Timothy Man-Yau Cheung, George Pak-Heng Leung

**Affiliations:** ^1^Department of Pharmacology and Pharmacy, Li Ka Shing Faculty of Medicine, The University of Hong Kong, Hong Kong SAR, China; ^2^Department of Rehabilitation Sciences, Faculty of Health and Social Sciences, Hong Kong Polytechnic University, Hong Kong SAR, China; ^3^State Key Laboratory of Southwestern Chinese Medicine Resources, School of Pharmacy, Chengdu University of Traditional Chinese Medicine, Chengdu, China; ^4^State Key Laboratory of Quality Research in Chinese Medicine and Institute of Chinese Medical Sciences, University of Macau, Macao SAR, China; ^5^Tian Ran Healthcare Limited, Hong Kong, China

## Abstract

Clinical outcomes for doxorubicin (Dox) are limited by its cardiotoxicity but a combination of Dox and agents with cardioprotective activities is an effective strategy to improve its therapeutic outcome. Natural products provide abundant resources to search for novel cardioprotective agents. *Ganoderma lucidum* (GL) is the most well-known edible mushroom within the *Ganodermataceae* family. It is commonly used in traditional Chinese medicine or as a healthcare product. *Amauroderma rugosum* (AR) is another genus of mushroom from the *Ganodermataceae* family, but its pharmacological activity and medicinal value have rarely been reported. In the present study, the cardioprotective effects of the AR water extract against Dox-induced cardiotoxicity were studied *in vitro* and *in vivo*. Results showed that both the AR and GL extracts could potentiate the anticancer effect of Dox. The AR extract significantly decreased the oxidative stress, mitochondrial dysfunction, and apoptosis seen in Dox-treated H9c2 rat cardiomyocytes. However, knockdown of Nrf2 by siRNA abolished the protective effects of AR in these cells. In addition, Dox upregulated the expression of proapoptotic proteins and downregulated the Akt/mTOR and Nrf2/HO-1 signaling pathways, and these effects could be reversed by the AR extract. Consistently, the AR extract significantly prolonged survival time, reversed weight loss, and reduced cardiac dysfunction in Dox-treated mice. In addition, oxidative stress and apoptosis were suppressed, while Nrf2 and HO-1 expressions were elevated in the heart tissues of Dox-treated mice after treatment with the AR extract. However, the GL extract had less cardioprotective effect against Dox in both the cell and animal models. In conclusion, the AR water extract demonstrated a remarkable cardioprotective effect against Dox-induced cardiotoxicity. One of the possible mechanisms for this effect was the upregulation of the mTOR/Akt and Nrf2/HO-1-dependent pathways, which may reduce oxidative stress, mitochondrial dysfunction, and cardiomyocyte apoptosis. These findings suggested that AR may be beneficial for the heart, especially in patients receiving Dox-based chemotherapy.

The article "Protective Effects of Amauroderma rugosum on Doxorubicin-Induced Cardiotoxicity through Suppressing Oxidative Stress, Mitochondrial Dysfunction, Apoptosis, and Activating Akt/mTOR and Nrf2/HO-1 Signaling Pathways" was retracted in 2023. Reasons: signs of a paper mill; compromised peer review; unreliable results or conclusions.

## 1. Introduction

Doxorubicin (Dox) is one of the most widely used and effective antineoplastic agents for the treatment of various types of cancer, including breast, ovarian, gastric, bladder, and thyroid cancers [1]. However, the cardiotoxicity of Dox limits its clinical applications [2]. Clinical studies have shown that the incidence of cardiotoxicity is approximately 5% when the cumulative dose of Dox is 400 mg/m^2^. However, this incidence can dramatically increase to 26% and 49% when the cumulative dose of Dox is 550 mg/m^2^ and 700 mg/m^2^, respectively [2]. The symptoms of Dox-induced cardiotoxicity include arrhythmia, cardiomyopathy, left ventricular dysfunction, and congestive heart failure [3]. Although the exact mechanisms involved in Dox-induced cardiotoxicity remain elusive, making it difficult to develop appropriate detoxification drugs [4], oxidative stress is considered to be its major causal factor [5]. Dox can stimulate the generation of excessive reactive oxygen species (ROS) in rat cardiomyocytes by increasing the accumulation of intracellular Ca^2+^ [6]. In clinical studies, oxidative stress was markedly increased in heart tissues when the cumulative dosage of Dox exceeded 500 mg/m^2^ [7].

Although oxidative stress is the most widely studied cause, accumulating evidence has indicated that a dysfunction in the nuclear factor erythroid 2-related factor 2 (Nrf2)/Heme oxygenase- (HO-) 1 pathway is also closely involved in the regulation of Dox-induced cardiotoxicity. Nrf2 is a transcription factor responsible for the regulation of cellular redox balance and protective antioxidant and phase II detoxification responses in mammals [8]. Under physiological conditions, Nrf2 combines with proteasomal degradation in the cytosol by the 26S proteasome via the cytoplasmic binding protein kelch-like epichlorohydrin-related protein (Keap) 1 [9]. However, under stressful conditions, Nrf2 is released from Keap1 and translocates to the nucleus. After binding to the antioxidant response element sequence, Nrf2 activates and upregulates the expression of downstream antioxidant proteins and biphasic detoxification enzymes, including HO-1, NAD(P)H:quinone oxidoreductase-1, and glutathione S-transferase, ultimately facilitating intracellular antioxidative responses [10]. It has been reported that the Nrf2-dependent antioxidant response system is suppressed in the hearts of Dox-treated rats, which is consistent with the observed decrease in protein abundance of Nrf2 [11]. Additionally, Dox-induced oxidative stress, cardiomyocyte necrosis, and cardiac dysfunction were found to be exaggerated in Nrf2 knockout mice [12]. Therefore, the Nrf2/HO-1 signaling pathway may be a potential drug target for the prevention and/or treatment of Dox-induced cardiotoxicity.

The article "Protective Effects of Amauroderma rugosum on Doxorubicin-Induced Cardiotoxicity through Suppressing Oxidative Stress, Mitochondrial Dysfunction, Apoptosis, and Activating Akt/mTOR and Nrf2/HO-1 Signaling Pathways" was retracted in 2023. Reasons: signs of a paper mill; compromised peer review; unreliable results or conclusions.

Natural products provide abundant resources for the discovery of novel cardioprotective agents. Our previous studies have demonstrated that oridonin [13] and glycyrrhetinic acid [14, 15] do not only enhance the anticancer efficacy of Dox in breast cancer but also show a potential positive activity in ameliorating Dox-induced cardiotoxicity. *Ganoderma lucidum* (GL), also known as “Lingzhi” in China, is one of the most well-known mushrooms and has been widely used in traditional Chinese medicine for centuries. A prior study has shown that GL extract can prevent Dox-induced cardiotoxicity by reducing Dox-induced oxidative stress in rats [16]. It has also been reported that GL polysaccharides can ameliorate Dox-induced mitochondrial damage, oxidative stress, proinflammatory cytokine production, and rat cardiomyocyte apoptosis. The underlying mechanism of GL polysaccharides is likely attributed to the rescue of the Nrf2/HO-1 signaling pathway, which is suppressed by Dox [17].

*Amauroderma rugosum* (AR) is another genus of basidiomycete within the *Ganodermataceae* family. Its cap is black in color and is irregularly wrinkled with thin or blunt edges. Its hymenium has a white surface, which turns dark red when scratched. Because of this, AR is also called “blood Linzhi” in Chinese [18]. AR has been used as a traditional medicine in China and Malaysia for the treatment of inflammation, cancers, gastric disorders, and epilepsy [19]. Although AR is consumed by people in China and South Asia, very few scientific studies have been conducted to explore its medicinal value or its beneficial effects on human health. We have previously reported that AR extract can protect PC12 neuroblastoma cells against 6-OHDA-induced toxicity through its antioxidant and antiapoptotic effects [18]. It has been hypothesized that AR may also influence reducing Dox-induced cardiotoxicity due to its remarkable antioxidant capacity. In the present study, the effect of AR extract on Dox-induced cardiotoxicity and its underlying cardioprotective mechanisms were investigated *in vitro* and *in vivo*, and its efficacy was also compared to that of GL.

The article "Protective Effects of Amauroderma rugosum on Doxorubicin-Induced Cardiotoxicity through Suppressing Oxidative Stress, Mitochondrial Dysfunction, Apoptosis, and Activating Akt/mTOR and Nrf2/HO-1 Signaling Pathways" was retracted in 2023. Reasons: signs of a paper mill; compromised peer review; unreliable results or conclusions.

## 2. Materials and Methods

### 2.1. Ethical Statement

Ethical research considerations were approved by the Chengdu University of Traditional Chinese Medicine. All experimental protocols using animals were conducted in compliance with guidelines established by the Institutional Animal Care and Use Committee (no. CDU2019S121), and animal welfare has been ensured throughout the animal experiments.

### 2.2. Materials

Dimethyl sulfoxide (DMSO), trypan blue, paraformaldehyde, 3-(4,5-dimethylthiazol-2-yl)-2,5-diphenyltetrazoliumbromide (MTT), ganoderic acid A, ganoderic acid G, lucidenic acid A, and ergosterol were purchased from Sigma-Aldrich (St. Louis, MO, USA). Dulbecco's Modified Eagle Medium, fetal bovine serum, 4′,6-diamidino-2-phenylindole dye (DAPI), dihydroethidium (DHE), fluorescein phalloidin dye, annexin-V-conjugated fluorescein isothiocyanate (FITC) dye, 5,5′,6,6′-tetrachloro-1,1′,3,3′-tetraethylbenzimidazolocarbocyanine iodide (JC-1) dye, propidium iodide (PI) dye, bicinchoninic acid assay (BCA) kit, phenylmethylsulphonyl fluoride, CM-H_2_DCFDA dye, MitoSOX Red, penicillin/streptomycin, protease inhibitor cocktail, 0.25% (*w*/*v*) trypsin containing 1 mM EDTA, and phosphate-buffered saline (PBS) were all purchased from Invitrogen (Carlsbad, CA, USA). Terminal deoxynucleotidyl transferase dUTP nick end labelling (TUNEL) and lactate dehydrogenase (LDH) assay kits were obtained from Roche (Basel, Switzerland). Primary antibodies against Nrf2 and Keap1 were obtained from Abcam (Cambridge, UK). Other primary antibodies and secondary antibodies were purchased from Cell Signaling Technology (Danvers, MA, USA).

### 2.3. Reflux Extraction of AR and GL

Fruiting bodies of AR and GL were provided by Mytianran Healthcare Limited (Hong Kong, China), which has been granted an organic crop production certificate by the Hong Kong Organic Resource Centre. The extraction method has been described previously [18]. All extracts were dissolved in water and concentrated in 80 mL with a rotary evaporator and stored at −20°C before use.

### 2.4. Determination of Total Phenolic Compound, Polysaccharide, Triterpene, and Protein Content

The extracts were filtered and evaporated using a water bath. The residue was dissolved in 5 mL of distilled water, followed by a slow addition of 30 mL of 95% ethanol with stirring, and the samples were shaken and kept at 4°C overnight. After centrifugation, the supernatant was collected for the measurement of total content of phenolic compounds, triterpenes, and proteins. The precipitate was dissolved in hot water in a total volume of 35 mL and kept at 4°C for the detection of the total polysaccharide content. The methodology for determination of total phenolic compound, polysaccharide, and triterpene content has been described previously [18]. Glucose (GE), gallic acid (GAE), and oleanolic acid (OA) were used as standards during the chemical analysis of the polysaccharides, phenolic compounds, and triterpenes, respectively.

The article "Protective Effects of Amauroderma rugosum on Doxorubicin-Induced Cardiotoxicity through Suppressing Oxidative Stress, Mitochondrial Dysfunction, Apoptosis, and Activating Akt/mTOR and Nrf2/HO-1 Signaling Pathways" was retracted in 2023. Reasons: signs of a paper mill; compromised peer review; unreliable results or conclusions.

To measure total protein content in the extracts, a 1 mL sample was added into 4 mL of biuret reagent, mixed, and incubated at room temperature for 30 min. Then, the absorbance at 540 nm was measured with a microplate absorbance reader, and bovine serum albumin (BSA) was used as the standard and results expressed as mg of bovine serum albumin equivalent per g (mg BSA/g).

### 2.5. High-Performance Liquid Chromatography (HPLC) Analysis of Ganoderic Acid A, Ganoderic Acid G, Lucidenic Acid A, and Ergosterol

HPLC analysis was conducted according to the method described previously [20]. Briefly, the HPLC analysis was performed using an UltiMate 3000 HPLC analysis system (Thermo-Fisher, Waltham, MA, USA) with a DAD 3000 detector, ternary pump of SR3000 Solvent Rack, WPS-3000SL autosampler, TCC-3000SD column temperature controller, and Chromeleon 7.2. Separation and was achieved in a C18 reversed-phase column (Hypersil Gold, particle size 5 *μ*m, 250 mm × 4.6 mm, Thermo Scientific). The mobile phase contained acetonitrile (solvent A) and 0.1% phosphoric acid aqueous solution (solvent B). The detailed gradient elution program was as follows: 0–25 min, 25–50% A; 25–30 min, 50–99% B; and 30–50 min, 99–99% B; and HPLC profiling was performed at 30°C at a constant flow rate of 1.0 mL/min. All samples were injected into the system at equal volumes of 10 *μ*L. Ganoderic acid A, ganoderic acid G, lucidenic acid A, and ergosterol were used as standards, and an analysis wavelength of 254 nm was selected.

### 2.6. Cell Culture

Rat cardiomyoblasts H9c2 and human breast adenocarcinoma cells MDA-MB-231 and MCF-7 were obtained from the American Type Culture Collection (Manassas, VA, USA) and cultured in Dulbecco's Modified Eagle Medium. The media was supplemented with 10% heat-inactivated fetal bovine serum and 1% penicillin/streptomycin. All cells were incubated at 37°C in a humidified atmosphere with 5% CO_2_.

### 2.7. Cell Viability Assay

Cell viability was measured with an MTT assay according to the manufacturer's protocol. Briefly, cell culture medium was replaced with MTT solution (0.5 mg/mL) after drug treatment, and the cells were incubated for an additional 4 h at 37°C. The MTT solution was then discarded, 100 *μ*L of DMSO was added to each well to dissolve the violet formazan crystals formed within the cells, and absorbance at 570 nm was measured with a SpectraMax M5 Multimode Microplate Reader (Molecular Devices, Sunnyvale, CA, USA).

The article "Protective Effects of Amauroderma rugosum on Doxorubicin-Induced Cardiotoxicity through Suppressing Oxidative Stress, Mitochondrial Dysfunction, Apoptosis, and Activating Akt/mTOR and Nrf2/HO-1 Signaling Pathways" was retracted in 2023. Reasons: signs of a paper mill; compromised peer review; unreliable results or conclusions.

### 2.8. LDH Assay

Cellular injury was assessed by measuring the activity of LDH released into the culture medium using a commercial kit (Roche, Basel, Switzerland) according to the manufacturer's instructions. Absorbances at 490 nm were measured on a microplate reader.

### 2.9. Seahorse Assay

Mitochondrial oxygen consumption rates (OCR) were measured using a Seahorse XFe24 Analyzer (Seahorse Biosciences, Billerica, MA, USA). H9c2 cells (8 × 10^3^ cells/well) were seeded into Seahorse XF 24 well culture microplates and incubated overnight at 37°C in a humidified atmosphere with 5% CO_2_. After drug treatment, the culture medium was replaced with Seahorse base medium and incubated in a non-CO_2_ incubator for 1 h. H9c2 cells were sequentially treated with 1 *μ*M oligomycin (Oligo), 5 *μ*M carbonyl cyanide-4-(trifluoromethoxy) phenylhydrazone (FCCP), and 1 *μ*M rotenone plus 1 *μ*M antimycin A (R + A). Then, OCR was calculated using Seahorse software (Seahorse Biosciences). After the assay was completed, the cells were lysed with radioimmunoprecipitation assay (RIPA) buffer (200 *μ*L/well), and the protein concentration was measured using the BCA and OCR values were normalized to the protein content and presented as pmol/min/*μ*g protein.

### 2.10. DAPI/Phalloidin and Annexin V/PI Double Staining

Apoptosis was assessed using DAPI/phalloidin and annexin V/PI double staining. H9c2 cells were seeded in 12-well plates (2 × 10^5^ cells/well) overnight and then treated with the appropriate drug. After, the cells were washed twice with ice-cold PBS and stained with DAPI (2.0 *μ*g/mL) and phalloidin-FITC (0.5 *μ*M) for 20 min at 37°C. Images were then captured using fluorescence microscopy (IN CELL Analyzer; GE Healthcare Life Sciences, Chicago, IL, USA). In addition, the H9c2 cells were harvested and resuspended in binding buffer and stained with annexin V-FITC and PI (1.0 mg/mL) for 15 min at 37°C. The stained cells were analyzed using a flow cytometer (BD Biosciences, San Jose, CA, USA) with 10 × 10^3^ events gated for each sample. The data were then analyzed using FlowJo software (BD Biosciences).

### 2.11. Measurement of Mitochondrial Membrane Potential

H9c2 cells were seeded overnight into 12-well plates (2 × 10^5^ cells/well); and after drug treatment, the cells were washed twice with warm PBS and stained with JC-1 dye (3 *μ*g/mL) for 20 min at 37°C. Images were then captured using a fluorescence microscope. In addition, the H9c2 cells were harvested and resuspended in warm PBS and then the cells were washed twice with warm PBS and examined using a flow cytometry.

The article "Protective Effects of Amauroderma rugosum on Doxorubicin-Induced Cardiotoxicity through Suppressing Oxidative Stress, Mitochondrial Dysfunction, Apoptosis, and Activating Akt/mTOR and Nrf2/HO-1 Signaling Pathways" was retracted in 2023. Reasons: signs of a paper mill; compromised peer review; unreliable results or conclusions.

### 2.12. ROS Detection

Intracellular and mitochondrial ROS were detected using CM-H_2_DCFDA and MitoSOX Red staining. After drug treatment, H9c2 cells were washed twice with cold PBS and stained with 2 *μ*M CM-H_2_DCFDA or MitoSOX Red for 15 min. After washing with PBS, a portion of the cells were imaged with a fluorescence microscope, and the remaining cells were harvested and analyzed using flow cytometry.

### 2.13. siRNA Knockdown of Nrf2

Nrf2 was knocked down specifically using siRNA as previously described [21]. H9c2 cells were transfected with either 100 nM Nrf2 siRNA or nontargeting scrambled siRNA (negative control) using Lipofectamine® 2000 reagent (Invitrogen; Carlsbad, CA, USA) for 24 h according to the manufacturer's protocol.

### 2.14. Western Blot Analysis

The western blot analysis methodology has been described previously [22]. Briefly, protein was extracted from H9c2 cells or mouse heart tissues with RIPA buffer containing 1% phenylmethylsulphonyl fluoride and 1% protease inhibitor. The cell lysate was then centrifuged for 20 min at 12,500 × *g* and 4°C to remove the nuclei and unbroken cells. The cytoplasmic and nuclear proteins were extracted using a nuclear and cytoplasmic protein extraction kit (Beyond time, Shanghai, China) according to the manufacturer's instructions. Protein concentrations were measured using BCAs. Equal amounts of protein were separated by electrophoresis using a sodium dodecyl sulphate–polyacrylamide gel and transferred to a polyvinylidene difluoride membrane (Bio-Rad Laboratories, Hercules, CA, USA). Nonspecific antigen binding was blocked with 5% nonfat milk for 1 h at room temperature. The membranes were then probed with primary antibodies against PARP, cleaved-PARP (Asp214), caspase 3, cleaved-caspase 3 (Asp175), caspase 9, cleaved-caspase 9 (Asp315), Bax, Bcl-2, mTOR, phospho-mTOR (Ser2448), Akt, phospho-Akt (Ser473), Nrf2, Keap1, HO-1, or *β*-actin overnight at 4°C. All primary antibodies were diluted at a ratio of 1 : 1,000 in Tris-buffered saline with 0.05% Tween 20 (TBST). After washing three times with TBST, the membranes were incubated with horseradish peroxidase-conjugated secondary antibodies (1 : 2,000 dilution in TBST) for 2 h at room temperature. After multiple washes with TBST, protein bands were developed using enhanced chemiluminescence. Images of the protein bands were captured, and densitometric measurements of signal intensities were collected with a chemiluminescence system (Syngene, Frederick, MD, USA). Protein expression of *β*-actin was similarly detected with a monoclonal mouse antiactin antibody (Chemicon, Temecula, CA, USA), and the optical density values for the different bands were normalized to those of *β*-actin.

The article "Protective Effects of Amauroderma rugosum on Doxorubicin-Induced Cardiotoxicity through Suppressing Oxidative Stress, Mitochondrial Dysfunction, Apoptosis, and Activating Akt/mTOR and Nrf2/HO-1 Signaling Pathways" was retracted in 2023. Reasons: signs of a paper mill; compromised peer review; unreliable results or conclusions.

### 2.15. Animal Study

Eight-week-old male C57BL/6 J mice (~25 g) were supplied by the animal centre of Sichuan Provincial Academy of Medical Sciences and kept under a 12 h light/dark cycle at the animal care facility with an ambient temperature controlled at 20 ± 5°C. The animals were fed with a fresh diet (containing 40% corn, 26% bran, 29% soybean cake, 1% salt, 1% bone meal, and 1% lysine) and had free access to water. The mice were acclimated for at least 7 days before the experiments and then divided into four groups (*n* = 8): (i) saline, (ii) Dox, (iii) Dox + AR, and (iv) Dox + GL. The sample size was calculated using the animal sample size calculator InVivoStat (with a power of 90%). The mice in the Dox + AR and Dox + GL groups were first administered AR (250 mg/kg) or GL (250 mg/kg) by oral gavage for 28 consecutive days. Starting from day 13, the mice received intraperitoneal injections of Dox (5 mg/kg) every 3 days until a cumulative dose of Dox (25-mg/kg) was reached to induce cardiotoxicity. The mice in the saline and Dox groups were treated with equal volumes of water for 28 days and received intraperitoneal injections of saline and Dox since day 13. The dose of DOX was chosen based on a previous report [5]. Regarding the dose of AR and GL, a previous report showed that treatment with 50 mg/kg of GL polysaccharide for 14 days had cardioprotective effect on Dox-treated rats [17]. Our chemical analysis showed that the polysaccharide content in AR and GL was approximately 5%, which suggested that 1000 mg/kg of AR and GL should be used. However, since the duration of treatment was 28 days instead of 14 days, the dose should be reduced. Our preliminary studies revealed that there was no significant difference between 250 mg/kg and higher doses in terms of the cardioprotective effect, and therefore, a dose of 250 mg/kg was used in the present study. Body weights and health of the animals were monitored every other day and the experiments would be stopped, and the animals would be removed from the study if they were unable to eat or drink, showed any abnormal behavior, or signs of toxicity, pain, or distress. At the end of the experiment, the mice were euthanized by an overdose of sodium pentobarbital (150 mg/kg), and death was confirmed by the absence of a heartbeat. Then, blood was collected for the assessment of cardiac injury by measuring serum LDH and creatine kinase (CK) levels. The heart tissues were excised, weighed, fixed with 4% (*v*/*v*) formaldehyde, dehydrated, and cut into 6 *μ*m sections. Then, tissue morphology, oxidative stress, and cell apoptosis were examined by hematoxylin and eosin, DHE, and TUNEL staining. In addition, the sections were immunostained with monoclonal antimouse Nrf2 and HO-1 antibodies to investigate the expression of Nrf2 and HO-1 in heart tissues.

The article "Protective Effects of Amauroderma rugosum on Doxorubicin-Induced Cardiotoxicity through Suppressing Oxidative Stress, Mitochondrial Dysfunction, Apoptosis, and Activating Akt/mTOR and Nrf2/HO-1 Signaling Pathways" was retracted in 2023. Reasons: signs of a paper mill; compromised peer review; unreliable results or conclusions.

### 2.16. Survival Rate Analysis

The mean survival time and percentage change in life span were calculated based on mortality of the experimental mice with Dox treatment (*n* = 8). All the animals were allowed a natural death, and animal survival rate was analyzed using a Kaplan-Meier method. Statistical differences were calculated with a log-rank test.

### 2.17. Echocardiography

To determine cardiac function, the mice were anesthetized with 1% isoflurane in O_2_ gas and then placed on a heated imaging platform. Echocardiographic experiments were performed using a Vevo 3100 microultrasound imaging system (Visual Sonics Inc., Toronto, Canada) equipped with a 15 MHz linear transducer. The parameters of left ventricular fractional shortening (LVFS) and left ventricular ejection fraction (LVEF) were analyzed using Vevo LAB software (FUJIFILM VisualSonics, Toronto, ON, Canada).

### 2.18. Biochemical Analysis

LDH and CK levels in the serum and malondialdehyde (MDA) levels, reduced glutathione (GSH) levels, superoxide dismutase (SOD) activity, and catalase (CAT) activity in the heart tissues were measured using commercial kits (Abcam, Cambridge, UK) following the manufacturer's instructions.

### 2.19. Statistical Analysis

Data were analyzed in Prism v.5.0 software (GraphPad, La Jolla, CA, USA) and expressed as the mean ± standard deviation (SD). The differences between groups were compared using one-way ANOVA, and *p* < 0.05 was considered to indicate statistically significant differences.

## 3. Results

### 3.1. Chemical Composition of AR and GL Extracts

Chemical assay results showed that the content of total polysaccharides in the AR and GL extracts was 42.45 ± 2.88 and 33.48 ± 2.97 mg GE/g, respectively. The content of total triterpenes included 6.10 ± 0.02 mg OA/g in the AR extract and 4.42 ± 0.134 mg OA/g in the GL extract. The content of total phenolic compounds was 6.60 ± 0.13 mg GAE/g in the AR extract and 3.68 ± 0.21 mg GAE/g in the GL extract. The content of total proteins in the AR and GL extracts was 212.01 ± 8.29 mg BSA/g and 160.02 ± 4.95 mg BSA/g, respectively (Table 1).

### 3.2. HPLC Analysis of the Major Components Found in AR and GL Extracts

The major components of the AR and GL extracts, including ganoderic acid A, ganoderic acid G, lucidenic acid A, and ergosterol, were quantified using HPLC. The results showed that the amount of ganoderic acid A and lucidenic acid A in the AR extract was lower than that in the GL extract, while the amount of ganoderic acid G and ergosterol in the AR extract was greater than that found in the GL extract (Figure S1). The average amount of ganoderic acid A, ganoderic acid G, lucidenic acid A, and ergosterol in the AR extract was 9.39, 12.20, 15.69, and 1477.68 *μ*g/g, respectively (Table 2). The average amount of ganoderic acid A, lucidenic acid A, and ergosterol in the GL extract was 41.73, 51.21, and 1070.23 *μ*g/g, respectively. However, ganoderic acid G could not be detected in the GL extract.

The article "Protective Effects of Amauroderma rugosum on Doxorubicin-Induced Cardiotoxicity through Suppressing Oxidative Stress, Mitochondrial Dysfunction, Apoptosis, and Activating Akt/mTOR and Nrf2/HO-1 Signaling Pathways" was retracted in 2023. Reasons: signs of a paper mill; compromised peer review; unreliable results or conclusions.

### 3.3. Effect of AR and GL Extracts on Dox-Induced Toxicity in H9c2 Cells

Cytotoxicity in H9c2 cells was evaluated using MTT and LDH assays, and the results showed that a 24 h treatment with Dox exhibited significant toxicity in H9c2 cells. Viability of H9c2 cells decreased by 54%, and LDH levels increased by 55% after treatment with Dox (Figures 1(a) and 1(b)). However, both the AR and GL extracts showed no toxicity in H9c2 cells at concentrations ranging from 0.125–2 mg/mL (data not shown). The AR extract increased cell viability and decreased LDH levels in a dose-dependent manner at concentrations ranging from 0.5–2 mg/mL in Dox-treated H9c2 cells. However, the GL extract had no effect (Figures 1(a) and 1(b)).

Seahorse assay was performed to evaluate mitochondrial function in H9c2 cells. After a 24 h treatment, Dox significantly induced mitochondrial dysfunction in H9c2 cells by markedly inhibiting basal respiration, ATP-linked respiration, maximal respiration, and spare respiration capacity (Figures 1(c)to 1(g)). By contrast, basal respiration, ATP-linked respiration, maximal respiration, and spare respiration capacity in Dox-treated cells after treatment with the AR extract were increased by 63%, 57%, 181%, and 67%, respectively. However, GL showed no effects on reducing Dox-induced mitochondrial dysfunction in H9c2 cells. In addition, MDA-MB-231 and MCF-7 human breast cancer cells were used to evaluate the impact of the AR and GL extracts on the anticancer effect of Dox. The results showed that both the AR and GL extracts significantly enhanced the anticancer effects of Dox in MDA-MB-231 and MCF-7 breast cancer cells (Figures 1(h) and 1(i)).

### 3.4. Effect of AR and GL Extracts on Dox-Induced Apoptosis in H9c2 Cells

A reduction in mitochondrial membrane potential (MMP) is an initial and irreversible step towards apoptosis. To evaluation of MMP, H9c2 cells were stained with JC-1 dye, and the changes in MMP were assessed using confocal microscopy and flow cytometry. The AR and GL did not affect MMP in H9c2 cells since no obvious green signals were observed. In contrast, Dox significantly induced the loss of MMP in H9c2 cells as reflected by the change from red to green fluorescence (Figures 2(a) and 2(b)). Quantitative analysis of microscopy images (Figure 2(e)) and flow cytometry (Figure 2(f)) showed that Dox decreased MMP in H9c2 cells by 77% and 48%, respectively. However, Dox-induced loss of MMP was remarkably rescued by the AR but not the GL extract. After AR extract treatment, the MMP from the Dox-treated H9c2 cells was only decreased by 41% and 2% in microscopy images and flow cytometry analysis (Figures 2(e) and 2(f)), respectively.

The article "Protective Effects of Amauroderma rugosum on Doxorubicin-Induced Cardiotoxicity through Suppressing Oxidative Stress, Mitochondrial Dysfunction, Apoptosis, and Activating Akt/mTOR and Nrf2/HO-1 Signaling Pathways" was retracted in 2023. Reasons: signs of a paper mill; compromised peer review; unreliable results or conclusions.

DAPI/phalloidin double staining was used to evaluate apoptosis in H9c2 cells, and no nuclear condensation or fragmentation was observed in the control, AR, and GL extract-treated cells. In contrast, many bright condensed dots that represent apoptotic bodies were clearly observed in Dox-treated H9c2 cells (Figure 2(c)). Quantitative analysis showed that the number of apoptotic cells was 3.9-fold higher after treatment with 0.5 *μ*M Dox, and 1.4- and 2.8-fold higher when the H9c2 cells were pretreated with the AR and GL extracts before Dox treatment (Figure 2(g)). The antiapoptotic effect of the AR extract on H9c2 cells was also studied using annexin V-FITC and PI staining and flow cytometry (Figure 2(d)). The number of apoptotic cells was 4.4-fold higher after the treatment with Dox, but 1.9-fold and 3.7-fold higher when the cells were pretreated with the AR and GL extracts before the Dox treatment (Figure 2(h)).

### 3.5. Effect of AR and GL Extracts on Proapoptotic Protein Expression in H9c2 Cells

Expression of proteins involved in the apoptotic signaling pathways in H9c2 cells was studied using western blot assays (Figure 3). In comparison with the control group, both the AR and GL extract groups showed a small decrease in the expression of cleaved PARP, cleaved caspase-3, and Bax/Bcl-2 ratio. After a 24 h treatment with Dox (0.5 *μ*M), the ratios of cleaved PARP/PARP, cleaved caspase-3/caspase-3, cleaved caspase-9/caspase-9, and Bax/Bcl-2 were markedly increased by 198%, 191%, 245%, and 78%, respectively. However, the Dox-induced the elevation of the ratios of cleaved PARP/PARP, cleaved caspase-3/caspase-3, cleaved caspase-9/caspase-9, and Bax/Bcl-2 were abolished by the AR extract. Dox increased the ratios of cleaved PARP/PARP, cleaved caspase-3/caspase-3, and cleaved caspase-9/caspase-9 by 84%, 51%, and 148% after the treatment with the GL extract, respectively. However, the GL extract had no effect on the Dox-induced Bax/Bcl-2 ratio.

The article "Protective Effects of Amauroderma rugosum on Doxorubicin-Induced Cardiotoxicity through Suppressing Oxidative Stress, Mitochondrial Dysfunction, Apoptosis, and Activating Akt/mTOR and Nrf2/HO-1 Signaling Pathways" was retracted in 2023. Reasons: signs of a paper mill; compromised peer review; unreliable results or conclusions.

### 3.6. Effect of AR and GL Extracts on Dox-Induced ROS Generation in H9c2 Cells

Intracellular and mitochondrial ROS accumulation in H9c2 cells were evaluated as shown by staining with DCFDA and MitoSOX fluorescence dyes. The fluorescence signals were detected by confocal microscopy and flow cytometry. The AR and GL extracts showed no effects on intracellular ROS (green fluorescence) or mitochondrial ROS (red fluorescence) generation in H9c2 cells (Figures 4(a)–4(d)). Intracellular ROS generation in H9c2 cells was stimulated to 162% and 466% by Dox (0.5 *μ*M) as determined by confocal microscopy and flow cytometry, respectively (Figures 4(e) and 4(f)). Similarly, mitochondrial ROS generation in H9c2 cells was elevated to 125% and 89% by Dox (0.5 *μ*M) as determined by confocal microscopy and flow cytometry, respectively (Figures 4(g) and 4(h)). The effect of Dox on intracellular and mitochondrial ROS generation was abolished by the AR extract but not the GL extract (Figures 4(e)–4(h)).

### 3.7. Effect of AR and GL Extracts on Akt/mTOR and Nrf2/HO-1 Signaling Pathways in H9c2 Cells

The Akt/mTOR and Nrf2/HO-1 signaling pathways play vital roles not only in maintaining cardiomyocyte survival but also in the regulation of cardiomyocyte apoptosis. The expression levels of phospho-Akt, Nrf2, and HO-1 in H9c2 cells were significantly increased by the AR and GL extracts, whereas phospho-mTOR and Keap1 were not affected (Figure 5(a)). Notably, a 24 h treatment with Dox (0.5 *μ*M) inhibited the ratio of p-Akt/Akt, p-mTOR/TOR, Nrf2, and HO-1 by 27%, 75%, 79%, and 67%, respectively, but significantly elevated Keap1 expression by 257% in H9c2 cells (Figures 5(b)–5(f)). After treatment with the AR extract, the ratio of p-Akt/Akt was not decreased, while the ratio of p-mTOR/mTOR and the expression of Nrf2 and HO-1 in Dox-treated cells were decreased by 52%, 28%, and 25%, respectively. In addition, Dox-induced Keap1 expression was increased by 58% after treatment with the AR extract. After treatment with the GL extract, the p-Akt/Akt ratio was not reduced, and Keap1 expression in the Dox-treated H9c2 cells was increased to 65%. No effect of the GL extract on the ratio of p-mTOR/mTOR and expression of Nrf2 and HO-1 was observed (Figures 5(b)–5(f)). Furthermore, protein expression of Nrf2 in the cytosol of H9c2 cells was dose-dependently decreased by the AR extract whereas the protein expression of Nrf2 in the nucleus was significantly elevated by the AR extract (Figures 5(g)–5(h)).

### 3.8. Effect of Nrf2 Knockdown on the Protective Effect of AR Extract against Dox-Induced Toxicity in H9c2 Cells

To further investigate the role of Nrf2 in the cardioprotective effects of AR extract against Dox-induced cardiotoxicity, Nrf2 expression was knocked down in H9c2 cells using siRNA transfection, and the protective effects of the AR extract were then examined. In comparison with the scramble siRNA-transfected cells, a mild decrease in cell viability and a slight increase in LDH release were observed in Nrf2 siRNA-transfected cells following Dox treatment (Figures 6(a) and 6(b)). AR extract (1 mg/mL) could alleviate Dox-induced cytotoxicity in the scramble siRNA-transfected cells, but it had no effect on Nrf2 siRNA-transfected H9c2s (Figures 6(a) and 6(b)). Similarly, knockdown of Nrf2 increased Dox-induced ROS generation and apoptosis in H9c2 cells (Figures 6(c)to 6(f)). AR could inhibit Dox-induced ROS generation and apoptosis in the scramble siRNA-transfected but not in Nrf2 siRNA-transfected cells (Figures 6(c)to 6(f)).

The article "Protective Effects of Amauroderma rugosum on Doxorubicin-Induced Cardiotoxicity through Suppressing Oxidative Stress, Mitochondrial Dysfunction, Apoptosis, and Activating Akt/mTOR and Nrf2/HO-1 Signaling Pathways" was retracted in 2023. Reasons: signs of a paper mill; compromised peer review; unreliable results or conclusions.

### 3.9. Effect of AR and GL Extracts on Protecting Dox-Induced Cardiotoxicity in Mice

A mouse model of Dox-induced cardiotoxicity was used to further investigate the cardioprotective effects of AR *in vivo*. A cumulative Dox dose of 25 mg/kg was injected into mice to induce cardiotoxicity. Dox induced a reduction in mouse body weight and an increase in the heart weight/body weight ratio (Figures 7(a) and 7(b)). The AR extract (250 mg/kg) alleviated the body weight loss and the increase in heart weight/body weight ratio in mice (Figures 7(a) and 7(b)). Additionally, the AR extract significantly prolonged the survival rate of Dox-treated mice (Figure 7(c)). Mouse cardiac functions were also evaluated using echocardiography (Figure 7(d)). Severe cardiac dysfunction was observed in the hearts of Dox-treated mice, with LVFS and LVEF decreased by 42% and 29%, respectively. Dox-induced cardiac dysfunction was markedly rescued by the AR extract, but not the GL extract. After treatment with the AR extract, LVFS and LVEF in Dox-treated mice were decreased by 8% and 5%, respectively (Figures 7(e) and 7(f)).

Next, myocardial injury was evaluated by analyzing cardiac damage markers, including LDH and CK. Dox treatment significantly increased the serum levels of LDH and CK in mice, and these effects were markedly reduced by the AR extract but not the GL extract (Figures 7(g) and 7(h)). MDA, SOD, GSH, and CAT levels in the heart tissues were also examined, and we found that MDA levels were elevated by Dox, whereas the increased MDA levels were significantly suppressed by the AR extract (Figure 7(i)). Moreover, SOD activity in the heart was slightly decreased by Dox but significantly elevated after treatment with the AR extract (Figure 7(j)). Furthermore, GSH and CAT activities in the heart were significantly inhibited by Dox, and this inhibition was abolished by AR treatment (Figures 7(k) and 7(m)). Although GL treatment slightly decreased MDA levels and increased SOD, GSH, and CAT activities in Dox-treated mice, the difference was not statistically significant. Western blot results for mouse heart tissues showed that the ratio of phosphor-Akt/Akt and expression levels of Nrf2 and HO-1 were decreased by Dox 58%, 48%, and 50%, whereas the Bax/Bcl-2 ratio and cleaved caspase-3/caspase-3 ratio were elevated by Dox to 643% and 204%, respectively, in the mouse heart tissues (Figure 7(l)). With AR extract treatment, the ratio of p-Akt/Akt and the expression of HO-1 could not be reduced, and the expression of Nrf2 could only be decreased by 23% (Figures 7(n)–7(p)). Moreover, the ratio of Bax/Bcl-2 and cleaved caspase-3/caspase-3 could only be increased by 230% and 14%, respectively (Figures 7(q) and 7(r)).

The article "Protective Effects of Amauroderma rugosum on Doxorubicin-Induced Cardiotoxicity through Suppressing Oxidative Stress, Mitochondrial Dysfunction, Apoptosis, and Activating Akt/mTOR and Nrf2/HO-1 Signaling Pathways" was retracted in 2023. Reasons: signs of a paper mill; compromised peer review; unreliable results or conclusions.

In addition, tissue morphology, ROS accumulation, apoptosis, and expression levels of Nrf2 and HO-1 in the mouse heart were examined using histological analyses. Cardiotoxicity was demonstrated in the Dox-treated mice based on the observation of fewer cardiomyocytes in the cardiac tissues and an increase in nuclear chromatin condensation in these cells (Figure 8(a)). Cardiotoxicity was reduced by the AR extract, but not the GL extract (Figure 8(a)). Dox also induced ROS accumulation and apoptosis in mouse hearts as the positive DHE and TUNEL signals were drastically increased (Figures 8(b) and 8(c)). The expression of Nrf2 and HO-1 in mouse hearts was also suppressed by Dox (Figures 8(d) and 8(e)). However, all the above effects induced by Dox could be reversed by the AR extract, but not the GL extract (Figures 8(f)–8(i)).

## 4. Discussion

Oxidative stress is considered to be one of the main causes of Dox-induced cardiac injury [23] as an imbalance between ROS and antioxidants can lead to oxidative stress [24, 25]. Sustained oxidative stress caused by Dox can reduce the mitochondrial membrane potential, which induces mitochondrial dysfunction and cell apoptosis and ultimately leads to cardiomyocyte damage [26]. Although the pharmacological effects of AR have rarely been investigated, AR extracts have been shown to inhibit oxidants and proinflammatory mediators such as TNF-*α* and nitric oxide in LPS-stimulated RAW264.7 cells [27, 28]. Moreover, AR extracts showed potential antioxidant and antiatherosclerotic effects in *in vivo* models by inhibiting low-density lipoprotein (LDL) level, LDL peroxidation, and 3-hydroxy3-methylglutaryl-coenzyme A (HMG-CoA) reductase catalytic activity [29]. Furthermore, a recent study indicated that ethanol extract of AR showed potential gastroprotective effects in rat gastric ulcer models by suppressing inflammation through the inhibition of NF-*κ*B and NLRP3 gene expression [30]. Our previous study has also demonstrated that AR possessed a remarkable ability to remove ROS and exhibited promising neuroprotective effects in PC12 cells by reducing 6-OHDA-induced oxidative stress, mitochondrial dysfunction, and apoptosis [18]. Although the above studies have suggested an antioxidant property of AR, and heart is well-known to be vulnerable to oxidative stress, the effect of AR on heart has not hitherto been explored. The present study is aimed at filling this research gap, and to our knowledge, we are the first to report that the AR extract could rescue cardiomyocytes from Dox-induced cell death by reducing Dox-induced oxidative stress, mitochondrial dysfunction, and apoptosis.

The article "Protective Effects of Amauroderma rugosum on Doxorubicin-Induced Cardiotoxicity through Suppressing Oxidative Stress, Mitochondrial Dysfunction, Apoptosis, and Activating Akt/mTOR and Nrf2/HO-1 Signaling Pathways" was retracted in 2023. Reasons: signs of a paper mill; compromised peer review; unreliable results or conclusions.

In terms of the mechanism of cardioprotective action, our results showed that the AR extract may activate the Akt/mTOR signaling pathway, which is known to play a vital regulatory role in cardiomyocyte survival [31]. Phosphorylation of Akt and mTOR was inhibited by Dox in H9c2 cells, but this inhibition could be restored by AR treatment. Moreover, Dox-induced expression of proapoptotic proteins, such as cleaved-PARP, cleaved caspase-3, cleaved caspase-9, and Bax, could be suppressed by the AR extract. Previous studies have also reported that Dox-induced cardiotoxicity is likely due to the downregulation of the Nrf2/HO-1 signaling pathway [11]. Consistently, our results showed that Dox suppressed the expression of Nrf2 and HO-1 in H9c2 cells and mouse heart tissues, and this downregulation of Nrf2 and HO-1 could be significantly restored by the AR extract. Furthermore, AR also promoted the translocation of Nrf2 from the cytoplasm into nucleus. In addition, the cardioprotective effects of the AR extract against Dox-induced cardiotoxicity was abolished when Nrf2 was knocked down by siRNA. Taken together, our findings suggested that the cardioprotective effect of the AR extract may be related to the activation of both Akt/mTOR and Nrf2/HO-1-mediated mechanisms. Both the Akt/mTOR and Nrf2/HO-1 signaling pathways play important roles in the regulation of cell survival and antioxidative responses in cardiomyocytes [31, 32] and disruption of the Akt/mTOR or Nrf2/HO-1 signaling pathway can induce apoptosis in cardiomyocytes [31, 33]. Interestingly, previous studies have indicated that Akt is the upstream regulator of the Nrf2/HO-1 pathway [34, 35]. Therefore, there should be connection of abnormal expression of different proteins between the Akt/mTOR and Nrf2/HO-1 signaling pathways, which is worth to studying in the future.

The article "Protective Effects of Amauroderma rugosum on Doxorubicin-Induced Cardiotoxicity through Suppressing Oxidative Stress, Mitochondrial Dysfunction, Apoptosis, and Activating Akt/mTOR and Nrf2/HO-1 Signaling Pathways" was retracted in 2023. Reasons: signs of a paper mill; compromised peer review; unreliable results or conclusions.

An interesting finding from our study relates to the comparison of cardioprotective effects between the GL and AR water extracts. Previous studies have reported the cardioprotective effects of GL against Dox-induced cardiotoxicity [16, 17], and the present results showed that AR exhibited a greater effect than GL at inhibiting Dox-induced oxidative stress, mitochondrial dysfunction, and cell apoptosis in H9c2 cells. In our animal studies, the AR extract significantly protected the mice from Dox-induced body weight loss, reduced survival rate, and cardiac dysfunction. In our biochemical analyses, the AR extract significantly reversed Dox-induced upregulation of LDH, CK, and MDA levels but downregulated SOD, GSH, and CAT activities. Similarly, in the western blot analysis, the AR extract significantly rescued p-Akt, Nrf2, and HO-1 expression and significantly abolished ROS generation, apoptosis, and proapoptotic protein expression the heart tissue. However, all these protective effects were not observed in GL-treated mice.

The differences in the chemical constituent of AR and GL may provide some hint as to why AR exhibits superior protective effects on Dox-induced cardiotoxicity. A wide variety of constituents, including glycoproteins, polysaccharides, triterpenoids, meroterpenoids, sesquiterpenoids, steroids, alkaloids, benzopyran derivatives, and benzoic acid derivatives, have been found in GL [36]. Among them, polysaccharides are the most abundant component in the water extract [37]. They contribute to the major biological activities and therapeutic effects of GL [38]. It has been reported that GL polysaccharides alleviate Dox-induced cardiotoxicity by reversing Dox-induced cardiomyocyte death, apoptosis, oxidative stress, and proinflammatory cytokine production [17]. Moreover, GL polysaccharides stabilize Nrf2 expression by suppressing Gul3-mediated K48-linked polyubiquitination of Nrf2, leading to HO-1 activation and inhibition of the NF-*κ*B signaling pathway [17]. In contrast to these studies, the present results showed that the GL extract was not particularly effective in alleviating Dox-induced cardiotoxicity. This was likely due to the insufficient content of polysaccharides in the water extract. The present data showed that the polysaccharide concentration was equivalent to 33.5 *μ*g/mL and 42.5 *μ*g/mL in the GL and AR extracts (1 mg/mL), respectively. The polysaccharide concentration in the GL extract was lower than the effective dose of polysaccharides (i.e., 50 *μ*g/mL) used in a previous study [17]. Another possibility for the increased potency of the AR extract on cardioprotection may be due to the higher content of triterpenes, phenols, and ergosterol, which are known antioxidants [26]. Interestingly, ganoderic acid G was found in the AR extract but not in the GL extract, and the biological activity of ganoderic acid G has rarely been studied and thus its contribution to cardioprotection warrants further investigation.

The article "Protective Effects of Amauroderma rugosum on Doxorubicin-Induced Cardiotoxicity through Suppressing Oxidative Stress, Mitochondrial Dysfunction, Apoptosis, and Activating Akt/mTOR and Nrf2/HO-1 Signaling Pathways" was retracted in 2023. Reasons: signs of a paper mill; compromised peer review; unreliable results or conclusions.

In clinical practice, there are two main strategies used to reduce Dox-induced cardiotoxicity: structural modification of Dox using chemical and pharmaceutical methods and pharmacological approaches using drug combinations [26]. Currently, drugs that have been approved for the prevention of Dox-induced cardiotoxicity are rare. Dexrazoxane is the only such cardioprotective agent approved by the U.S. Food and Drug Administration and the European Medicines Agency (EMA) [39]. However, some severe deficiencies have led to restrictions on the use of dexrazoxane in the U.S. and some European countries [40]. As emerging evidence has suggested that dexrazoxane may significantly decrease the response rate of patients with advanced breast cancer receiving Dox treatment [41]. Moreover, dexrazoxane has carcinogenic potential, and its use shows an increased risk of developing acute myeloid leukemia and myelodysplastic syndrome [42]. Hence, dexrazoxane is contraindicated in children in Europe, and the EMA recommends that the use of dexrazoxane should be restricted in adult patients with advanced or metastatic breast cancer with a high risk of heart failure due to previous receipt of a high cumulative dose of Dox.

Discovery and development of novel drugs that can prevent Dox-induced cardiotoxicity will be of great value in clinical practice. Accumulating evidence has suggested that some natural products, including resveratrol [43], epigallocatechin-3-gallate [44], tanshinone IIA [45], and cardamonin [46], exhibit a remarkable ability to reduce Dox-induced cardiotoxicity. In addition, herbal extracts, including GL [17], *Ginkgo biloba* [47], and *Glycyrrhiza uralensis* [48], have also been demonstrated to possess significant cardioprotective effects against Dox-induced toxicity *in vitro* and *in vivo*. The present study demonstrated that AR extract not only enhanced the anticancer effects of Dox in breast cancer cells but also showed remarkable cardioprotective effects against Dox-induced cardiotoxicity. Therefore, further study on the potential application of AR or its active ingredients in chemotherapy is of great value.

## 5. Conclusions

In conclusion, the present study demonstrated that AR extract potentiated the cancer effect of Dox and was also a promising protective agent against Dox-induced cardiotoxicity by reducing oxidative stress, mitochondrial dysfunction, and cell apoptosis. The underlying mechanisms for this effect may involve the rescue of the Akt/mTOR and Nrf2/HO-1 signaling pathways. The cardioprotective activity of the AR extract was greater than that of the GL extract, and this was likely due to its higher polysaccharide, triterpene, polyphenol, ganoderic acid G, and ergosterol content. These findings provided valuable information for the future development of AR extracts and their active ingredients for use as a potential adjunct for Dox-based chemotherapy.

The article "Protective Effects of Amauroderma rugosum on Doxorubicin-Induced Cardiotoxicity through Suppressing Oxidative Stress, Mitochondrial Dysfunction, Apoptosis, and Activating Akt/mTOR and Nrf2/HO-1 Signaling Pathways" was retracted in 2023. Reasons: signs of a paper mill; compromised peer review; unreliable results or conclusions.

## Figures and Tables

**Figure 1:** Effect of AR and GL extracts on Dox-induced toxicity and mitochondrial dysfunction in H9c2 cells and the anticancer effect of Dox. H9c2 cells were pretreated with various concentrations of AR or GL extracts (0.125–2 mg/mL) for 12 h and then received a 0.5 *μ*M Dox treatment for a further 24 h. Cell viability and LDH release in H9c2 cells were examined by (a) MTT and (b) LDH assays. (c) Mitochondrial oxygen consumption rate (OCR) was monitored using a Seahorse metabolic analyzer. H9c2 cell response after addition of 1 *μ*M oligomycin (Oligo), 5 *μ*M FCCP, and 1 *μ*M rotenone plus 1 *μ*M antimycin (R + A) were recorded. (d) Basal respiration, (e) ATP-linked respiration, (f) maximal respiration, and (g) spare respiratory capacity in H9c2 cells were quantified. (h) MDA-MB-231 and (i) MCF-7 human breast cancer cells were treated with various concentrations of Dox (0–1 *μ*M) in the absence or presence of AR or GL (1 mg/mL) extracts for 48 h. Cell viability was measured using MTT assay, and data are presented as percentage of control group values (mean ± SD of three independent experiments). ^∗^*p* < 0.05 indicates a statistically significant difference.

**Figure 2:** Effect of AR and GL extracts on Dox-induced loss of mitochondrial membrane potential and apoptosis in H9c2 cells. H9c2 cells were pretreated with 1 mg/mL of AR or GL extract or vehicle (control) for 12 h and then treated with or without 0.5 *μ*M Dox for 24 h. (a) Mitochondrial membrane potential in H9c2 cells was then detected using fluorescence microscopy after JC-1 staining. Red and green fluorescence signals indicated JC-1 aggregates (which refers to the loss of mitochondrial membrane potential) and monomers, respectively. Scale bar: 100 *μ*m. (b) Flow cytometry analysis of mitochondrial membrane potential in H9c2 cells after JC-1 staining. The mitochondrial membrane potential in (e) microscopy images and (f) flow cytometry was quantified. (c) Apoptotic cells were detected by DAPI/phalloidin-FITC double staining. Blue and green signals show nuclei and cytoskeleton of H9c2 cells. White arrows indicate apoptotic cells, and the number of apoptotic cells was counted. Scale bar: 100 *μ*m. (d) Cells were double stained by annexin V-FITC and PI for 20 min and then analyzed using flow cytometry. The number of apoptotic cells in microscopy images (g) and flow cytometry (h) was quantified. Data are presented as percentage of control group values (mean ± SD of three independent experiments). ^∗^*p* < 0.05 indicates a statistically significant difference.

The article "Protective Effects of Amauroderma rugosum on Doxorubicin-Induced Cardiotoxicity through Suppressing Oxidative Stress, Mitochondrial Dysfunction, Apoptosis, and Activating Akt/mTOR and Nrf2/HO-1 Signaling Pathways" was retracted in 2023. Reasons: signs of a paper mill; compromised peer review; unreliable results or conclusions.

**Figure 3:** Effect of AR and GL extracts on Dox-induced expression of proapoptotic proteins in H9c2 cells. H9c2 cells were pretreated with 1 mg/mL of AR or GL extract or vehicle (control) for 12 h and then treated with or without Dox (0.5 *μ*M) for 24 h. Protein expression levels of PARP, cleaved-PARP, caspase-3, cleaved caspase-3, caspase-9, cleaved caspase-9, Bax, Bcl-2, and *β*-actin were examined using western blot analysis. (a) Representative blots. (b–d) Quantitative analysis of the ratios of protein expression level of (b) cleaved PARP/PARP, (c) cleaved caspase-3/caspase-3, (d) cleaved caspase-9/caspase-9, and (e) Bax/Bcl-2. Data are presented as percentage of control group values (mean ± SD of three independent experiments). ^∗^*p* < 0.05 indicates a statistically significant difference.

**Figure 4:** Effect of AR and GL extracts on Dox-induced oxidative stress in H9c2 cells. H9c2 cells were pretreated with 1 mg/mL of AR or GL extract or vehicle (control) for 4 h and then treated with or without 0.5 *μ*M Dox for 4 h. (a) Intracellular ROS and (b) mitochondrial ROS generation in H9c2 cells were detected by fluorescence microscopy after CM-H2DCFDA and MitoSOX red staining. Blue, green, and red signals indicate nuclei, intracellular ROS, and mitochondrial ROS in the H9c2 cells. Scale bar: 100 *μ*m. Flow cytometry analysis of (c) intracellular ROS and (d) mitochondrial ROS levels in H9c2 cells. Quantitative analysis of (e) intracellular ROS and (g) mitochondrial ROS levels using fluorescent microscopy. (f) Intracellular ROS and (h) mitochondrial ROS levels were quantified using flow cytometry analysis. Data are presented as percentage of control group values (mean ± SD of three independent experiments). ^∗^*p* < 0.05 indicates a statistically significant difference.

**Figure 5:** Effect of AR and GL extracts on the Akt/mTOR and Nrf2/HO-1 signaling pathways in H9c2 cells. H9c2 cells were pretreated with 1 mg/mL of AR or GL extract or vehicle (control) for 12 h and then treated with or without 0.5 *μ*M Dox for 24 h. (a) Protein expression levels of p-Akt, Akt, p-mTOR, mTOR, total Nrf2, Keap1, HO-1, and *β*-actin were examined using western blot analysis. (b)–(f) Quantitative analysis of protein expression levels. (g) H9c2 cells were pretreated with 0.5 and 1 mg/mL of AR for 12 h, and the protein expression levels of Nrf2 in the nucleus and cytosol were examined by western blot analysis. (h) Quantitative analysis of nuclear and cytosolic Nrf2 expression levels. Data are presented as percentage of control group (mean ± SD of three independent experiments). ^∗^*p* < 0.05 indicates a statistically significant difference.

The article "Protective Effects of Amauroderma rugosum on Doxorubicin-Induced Cardiotoxicity through Suppressing Oxidative Stress, Mitochondrial Dysfunction, Apoptosis, and Activating Akt/mTOR and Nrf2/HO-1 Signaling Pathways" was retracted in 2023. Reasons: signs of a paper mill; compromised peer review; unreliable results or conclusions.

**Figure 6:** Effect of Nrf2 knockdown on the protective effect of AR extract against Dox-induced toxicity in H9c2 cells. The H9c2 cells were transfected with scramble siRNA or siRNA against Nrf2 and pretreated with AR extract (1 mg/mL) or vehicle control (0.1% DMSO) for 12 h and then received a 0.5 *μ*M Dox treatment for an additional 24 h. Cell viability and LDH levels in the transfected H9c2 cells were examined by (a) MTT and (b) LDH assays. (c) Intracellular ROS generation in H9c2 cells was detected by flow cytometry after CM-H_2_DCFDA staining. (d) Cell apoptosis in H9c2 cells was detected using flow cytometry after annexin V-FITC and PI double staining. Quantitative analysis of (e) intracellular ROS levels and (f) apoptosis in transfected H9c2 cells. Data are presented as percentage of control group values (mean ± SD of three independent experiments). ^∗^*p* < 0.05 indicates a statistically significant difference and n.s. means not significant.

**Figure 7:** Effect of AR and GL extracts on Dox-induced cardiotoxicity in mice. Mice received AR (250 mg/kg) or GL (250 mg/kg) by oral gavage for 28 consecutive days. From day 13, the mice received intraperitoneal injection of Dox (5 mg/kg) every 3 days until a cumulative 25-mg/kg dose of Dox was reached that induced cardiotoxicity. Mice receiving vehicle (instead of AR or GL extract) and saline (instead of Dox) served as the control group. (a) Body weight was monitored every other day during the experimental period. (b) The ratio of heart weight to body weight was determined at the end of the experiment. (c) Kaplan-Meier survival curves for each group (*n* = 8) were monitored during the experiment. Statistical differences (*p* < 0.01) were calculated using the log-rank test. (d) Cardiac function in mice was evaluated as shown by echocardiography. Quantitative analysis of (e) left ventricular fractional shortening (LVFS) and (f) left ventricular ejection fraction (LVEF). (g) LDH and (h) CK activity in mouse serum was measured and quantified. (i) MDA, (j) SOD, (k) GSH, and (m) CAT levels in heart tissues were quantified. (l) Expression levels of p-Akt, Akt, total Nrf2, HO-1, Bax, Bcl-2, caspase-3, cleaved caspase-3, and GAPDH (as internal reference) in heart tissues were detected using western blot analysis. Quantitative analysis of the ratio of protein expression of (n) p-Akt/Akt, (o) Nrf2/GAPDH, (p) HO-1/GAPDH, (q) Bax/Bcl-2, and (r) cleaved caspase 3/caspase-3. Data are presented as percentage of control group values (mean ± SD of three independent experiments). ^∗^*p* < 0.05 indicates a statistically significant difference.

The article "Protective Effects of Amauroderma rugosum on Doxorubicin-Induced Cardiotoxicity through Suppressing Oxidative Stress, Mitochondrial Dysfunction, Apoptosis, and Activating Akt/mTOR and Nrf2/HO-1 Signaling Pathways" was retracted in 2023. Reasons: signs of a paper mill; compromised peer review; unreliable results or conclusions.

**Figure 8:** Histological analysis of heart tissues in the mouse model. Heart tissue samples (*n* = 8) were fixed with 4% (*v*/*v*) formaldehyde and cut into 6 *μ*m sections. (a) Sections were stained with hematoxylin and eosin to evaluate tissue architecture. Black arrows indicate lesions in the heart tissues. Sections were also stained with (b) DHE and (c) TUNEL to investigate ROS accumulation and apoptosis in heart cells, respectively. Sections were labeled with (d) anti-Nrf2 and (e) anti-HO-1 antibodies to evaluate oxidative stress in heart tissues. Red and green signals represent positive signals. Blue signals indicate cell nuclei inside the heart tissues. Scale bar: 100 *μ*m. Quantitative analysis of (f) DHE, (g) TUNEL, (h) Nrf2, and (i) HO-1 signals in heart tissues. Data are presented as the percentage of control (saline) group (mean ± SD of three independent experiments). ^∗^*p* < 0.05 indicates a statistically significant difference.

**Table 1:** Analysis of chemical content in AR and GL extracts.

Sample	Polysaccharides (mg GE/g)	Triterpenes (mg OA/g)	Phenols (mg GAE/g)	Proteins (mg BSA/g)
AR	42.45 ± 2.88	6.10 ± 0.02	6.60 ± 0.13	212.01 ± 8.29
GL	33.48 ± 2.97	4.42 ± 0.134	3.68 ± 0.21	160.02 ± 4.95

**Table 2:** HPLC analysis of the major components found in AR and GL extracts.

Sample	Ganoderic acid A (*μ*g/g)	Ganoderic acid G (*μ*g/g)	Lucidenic acid A (*μ*g/g)	Ergosterol (*μ*g/g)
AR	9.39	12.20	15.69	1477.68	
GL	41.73	Undetected	51.21	1070.23	

## Data Availability

The data that support the findings of this study are available from the corresponding author, George Pak-Heng Leung, upon reasonable request.

## Supplementary Materials

Supplementary Materials Figure S1: HPLC chromatograms of major components in AR and GL extract. (a) Mixed reference substances. (b) AR extract sample. (c) GL extract sample. Peak 1: ganoderic acid G; peak 2: ganoderic acid A; peak 3: lucidenic acid A; peak 4: ergosterol.
